The article "Industrial Internet of Things Model Driven by Particle Filter and Network Communication Technology" was retracted in 2023. Reasons: signs of a paper mill; suspected computer-generated content; unreliable results or conclusions; concerns about the data.

# Industrial Internet of Things Model Driven by Particle Filter and Network Communication Technology

**DOI:** 10.1155/2022/9026017

**Published:** 2022-07-14

**Authors:** Jianlan Liu

**Affiliations:** School of Electronic Information Engineering, Nantong Vocational University, Nantong, Jiangsu 226007, China

## Abstract

In this paper, a better particle filter algorithm is put forth to address the issues of particle filter sample exhaustion and weight degradation. The algorithm frames the received signal and separates the signals in two steps based on the slow-varying properties of system parameters in practical applications, such as phase shift and transmission delay. In addition, the network model and energy consumption model are built while the sensor data is being collected and processed using the industrial IoT's communication mechanism and algorithm. The repeater is chosen as the node with the lowest transmission energy consumption, and the industrial field's sensor data is gathered via the fog server node. The simulation results demonstrate that the proposed algorithm's accuracy rate is 95.54 percent, higher than that of the comparison algorithm. The enhanced algorithm suggested in this paper can simultaneously achieve improved parameter estimation performance and achieve signal separation with low bit error rates. Additionally, the communication system and algorithm can efficiently gather the sensing information from the industrial field, and the indicators like energy consumption and the first dead node are better than other algorithms. It offers an innovative method for enhancing industrial field application.

## 1. Introduction

A new kind of network known as the Internet of Things (IoT) uses information sensors to gather data about products and share that data with Internet resources in accordance with established rules. This network has made it possible to identify, monitor, transport, and control products. In order to achieve the goal of managing and controlling the IoT terminals, the IoT should enable remote monitoring and management, tracking and positioning, and on-site data collection and measurement. IoT communication has been used in the construction of the medical, aviation, military, agricultural, and other industries thanks to its advantages of convenience, strong robustness, and low cost. At the moment, with the rapid development of computer technology and communication [1, 2], the Industrial Internet of Things (IIoT) is a key technology for creating “smart businesses” and “smart industries” and has a broad range of potential applications in the industrial sector. IoT technology's application layer is where its primary growth and development are being driven by [3]. By implementing wireless sensor networks, the capabilities of the sensing layer and network layer can be realised. The field of intelligent industry has used wireless sensor networks extensively as a common data acquisition technique. The Internet of Things (IoT) is an extension of the Internet, so it is connected to many of the current network configurations [4]. Because it is a part of the network, the network is typically divided into several levels, with each level having its own functions and performance standards. The Internet of Things (IoT) technology is currently used to some extent in the industrial sector, but in actual use, its drawbacks—such as its enormous number of nodes and high levels of information redundancy—are in stark contrast to the energy resources available [4]. Studying the communication mechanism of the industrial IoT is of great practical significance because, at the same time, the traditional cloud architecture struggles with high network load and long end-to-end delays [5].

The article "Industrial Internet of Things Model Driven by Particle Filter and Network Communication Technology" was retracted in 2023. Reasons: signs of a paper mill; suspected computer-generated content; unreliable results or conclusions; concerns about the data.

Particle filtering has received extensive research as a nonlinear filtering technology in areas such as target tracking, visual tracking, robot positioning, wireless communication, and others [6]. Particle filter applications in signal processing can be categorised into two groups: multiple access systems and single-user systems. Because nonlinear and non-Gaussian tracking issues dominate the field of target tracking in the modern era, and because particle filter technology has excellent processing power for this model, it has garnered interest. The accuracy of intelligent monitoring is increased through the use of communication technology and information processing techniques, among which effective defence against the impact of unexpected information on network terminals is a key component [7]. Particle filter has grown in significance as the primary technique for state estimation in nonlinear and non-Gaussian dynamic systems. The algorithm removes the requirement that the random state variables must have previously satisfied the Gaussian distribution and is more accurate when dealing with the state estimation of nonlinear and non-Gaussian systems. Compared to the Gaussian model, it can express a wider range of arbitrary distributions and is better able to process state variable parameters with nonlinear properties [8]. Particle filter, which has no limitations on the system model or noise types, breaks through the Kalman filter's model framework at the same time and has a filtering accuracy that is close to optimal estimation. It can approximate the Bayesian estimation of the system by forecasting and updating the sampling set of the probability density function of the system. Particle filter offers a powerful remedy for the numerous nonlinear and non-Gaussian signal processing issues that contemporary communication faces [9]. There are still many issues to be solved, and the development of particle filters is not yet at a mature enough stage. Weight degradation and sample depletion are the two main drawbacks of particle filters. Weight degradation and sample depletion remain serious issues, despite the fact that there are numerous methods for solving these issues. This paper attempts to address this issue by enhancing particle filter and applying it to the industrial IoT's communication system. This paper investigates the industrial IoT's communication mechanism and algorithm based on particle filters. Its innovations are as follows: (1) Time-varying multiuser detection based on particle filter algorithm is studied in this paper. Aiming at the problem of large computation of particle filter, the particle filter is improved, and a separation algorithm based on dynamic particle filter is proposed. At the same time, from the perspective of differential evolution algorithm, by introducing adaptive strategy, the diversity of the sampled particles is increased by using adaptive differential mutation and adaptive differential hybridization, and then the problem of sample exhaustion caused by resampling is solved. (2) This paper analyzes the architecture of the IoT in detail and the network requirements of each layer. According to the typical application of IoT, the IoT system is classified and analyzed according to the carrying business. The communication mechanism and algorithm of industrial IoT are used to collect and process the sensing data, and the network model and energy consumption model are constructed. The node with the lowest transmission energy consumption is selected as the repeater, and the sensor data of the industrial field is collected through the fog server node. The experimental results show that it is effective and practical to apply the particle filter algorithm in industrial IoT communication.

The article "Industrial Internet of Things Model Driven by Particle Filter and Network Communication Technology" was retracted in 2023. Reasons: signs of a paper mill; suspected computer-generated content; unreliable results or conclusions; concerns about the data.

## 2. Related Work

The problem of filtering is how to restore the real signal from the observed signal polluted by noise. This kind of problem widely exists in engineering fields such as communication, signal processing, and target tracking, and the essence of filtering is statistical estimation. It is significant to study the communication mechanism of industrial IoT based on particle filter. Many scholars have studied it. With the continuous development of particle filter technology, the increasing complexity of system model in modern communication, and the increasing requirement of signal processing accuracy, particle filter will be applied more and more widely in communication signal processing.

Hai et al. proposed an improved hybrid Kalman filter algorithm. The method is as follows: first, the exact expression of the posterior distribution of the nonlinear state variable is obtained by recursion; then the *M* items with the largest weight are selected to approximate the real distribution; finally, the channel fading coefficient and transmission are estimated based on the approximate expression of the posterior distribution [10]. Hossain et al. pointed out that, in order to ensure the security of the IoT data fusion process, it is necessary to build a security data fusion method for the industrial IoT based on a supervision mechanism. Only in this way can the data fusion function be brought into full play and promote the improvement of the performance of the industrial IoT [11]. In order to obtain the posterior probability density function of the dynamic system state, Shin P J et al. used the sequential importance sampling technique to obtain a set of particles in the state space for the problem that multiple integrals cannot be calculated in Bayesian filtering. The set is substituted into the Bayesian estimation formula for iterative operation, and the corresponding weight of each particle is obtained; finally, the posterior probability density function of the state is approximated by the weighted summation of these particles [12]. Hybrid Kalman filter proposed by Xu et al. is a special case of particle filter dimensionality reduction technique [13]. The algorithm can solve the joint estimation problem of linear and nonlinear state variables. The variables are estimated using Kalman filtering. Lade et al. studied the blind separation of single-channel cochannel signals based on particle filtering. This system model also considers uncertain factors such as channel fading, timing deviation, frequency deviation, and phase deviation; the blind separation problem is transformed into a joint estimation problem of unknown parameters and information symbols, and the estimation is realised by particle filter algorithm [14]. Tang et al. proposed that the bearer network of the IoT requires more carrier-class features and puts forward high requirements for network service quality, security, and controllability. In order to meet the bearing of IoT services, it is necessary to further improve the carrier-class requirements of access networks, metropolitan area networks, and backbone networks, including end-to-end service quality capabilities, network self-healing capabilities, service protection capabilities, and network security [15]. In order to ensure the security of the data fusion process in the industrial IoT, Engel et al. proposed a security data fusion method for the industrial IoT based on a supervision mechanism [16]. Chen et al. used the Stiefel manifold model to describe the prior probability density and likelihood probability density of the state with the Langevin distribution and Gaussian distribution, respectively, and then updated the particles by sampling on the manifold distribution and then proposed the A particle filter algorithm based on Stiefel manifold [17]. Schraefel et al. believe that when the current method is used to balance the scheduling of nodes, the relationship between the remaining energy of the node and the energy consumption required for perception cannot be calculated, and there is a problem of low node scheduling accuracy. Therefore, a balanced scheduling method for target tracking nodes in IoT communication based on particle swarm is proposed [18]. Phan et al. used particle filtering for cooperative communication technology in wireless sensor networks, etc. [19].

The article "Industrial Internet of Things Model Driven by Particle Filter and Network Communication Technology" was retracted in 2023. Reasons: signs of a paper mill; suspected computer-generated content; unreliable results or conclusions; concerns about the data.

This paper provides a detailed analysis of the IoT architecture and network requirements for each layer based on related research. IoT systems are categorised and analyzed in accordance with the carrying business according to the typical application of the IoT. In a dynamic environment, blind separation of chaotic signals based on particle filters is also being researched. The particle filter algorithm is then used to track the number of active signals and realise the separation of chaotic signals in this paper. The random set model is used to fit the time-varying situation of the number of source signals. Additionally, from the perspective of the differential evolution algorithm, the problem of sample exhaustion brought on by resampling is resolved by introducing adaptive strategy, which increases the diversity of the sampled particles through the use of adaptive differential mutation and adaptive differential hybridization. The results of the experiment further support the viability and efficacy of using the particle filter algorithm in industrial IoT communication.

## 3. Methodology

### 3.1. Research on Communication Mechanism of Industrial IoT

With the rapid development of sensor technology, the IoT has been widely used in various fields [20]. The IoT is a kind of network that connects any required terminals to the Internet through radio frequency identification or various sensors and shares and exchanges data. The IoT also belongs to the Internet in essence, which is an extension and expansion of the Internet field. As a complex system that connects things and integrates various sensing devices and transmission devices, the IoT has formed its own unique architecture. In the future communication, the data traffic brought by the IoT will account for a large proportion of the total data traffic. Therefore, it will have an important impact on the carrying flow and the carrying mode of the communication network or the Internet. Generally, for the sake of simplicity, we model the wireless communication system as a linear Gaussian system, which is unfavorable to improve the data transmission quality of the wireless communication system in practical engineering applications. The actual wireless communication signal processing is to process the signals of nonlinear and non-Gaussian systems. The important functions of the IoT mainly include: (1) Perception of goods and information collection. (2) Transmission and sharing of information. (3) Effective supervision and intelligent handling of goods. The structure of the IoT can be divided into three levels from top to bottom: perception layer: perception layer is composed of various sensor nodes, which is used to collect the lowest sensor data. The main task of the sensing layer is to realise the intelligent sensing function and transform all kinds of physical quantities that need to be collected and monitored into digital information that can be processed in real time through corresponding technologies and equipment. Network layer: The function of the network layer is to send the control information of the application layer to the perception layer and transmit the data collected by the perception layer to the application layer. The network layer realises the connection between things and people. Application layer: The main purpose of the rise and development of IoT technology lies in the application layer. The main task of the application layer is to receive, analyze, and model all kinds of information and data from the network and then carry out the processing actions required by the system or extract useful information according to this information. The application layer realises man-machine interaction.  Figure 1 shows the layering and application model of the IoT.

The article "Industrial Internet of Things Model Driven by Particle Filter and Network Communication Technology" was retracted in 2023. Reasons: signs of a paper mill; suspected computer-generated content; unreliable results or conclusions; concerns about the data.

The amount of data is also growing exponentially along with the IoT access devices' explosive growth. The traditional centralised cloud architecture has issues with a high network load and a lengthy end-to-end delay. Due to this, it is essential to introduce data fusion technology in order to redundantly process the data already present in the industrial IoT, in order to increase data collection efficiency and reliability and conserve network energy. Sensors gather hundreds of billions of pieces of data simultaneously in IoT applications, which places high demands on the platform's capacity for data storage, aggregation, analysis, backup, and large-scale parallel computing. The Internet of Things (IoT) data acquisition system can establish a control centre that compiles data from various sensors and sends it all to a cloud calculator. Cloud computing can serve as the IoT's network engine by combining software operation, hardware operation, and virtualization to provide the best possible storage and computing capabilities. The main goals of wireless communication's future development are to expand voice, data, and bandwidth services. As a result, wireless communication systems will need to meet higher standards for data transmission rate, system performance, and system capacity. The design principle of the whole system of the IoT is not only to consider that the technology can be forward-looking, but also to ensure reliability, safe functions, and high performance. In order to ensure the future upgrade and expansion, the system should be well expandable. In order to meet the strict service quality requirements related to real-time IoT applications and maximize the overall efficiency, the cloud architecture is becoming more and more decentralized, and there are small cloud nodes at the edge of the network, such as fog nodes, thus forming the prototype of IoT communication mechanism with fog architecture. The distributed structure based on network control is a commonly used structure type in the IoT system. This type supports the network as the core, maintaining and scheduling all the acquisition devices, network devices, and scheduling devices in the IoT system.

All kinds of industrial sensor nodes form a large wireless sensor network, and the nodes in the wireless sensor network that can communicate with each other form independent subnets. The sensor nodes between subnets cannot transmit information to each other because the distance between them exceeds the communication range. Multicomponent mixed signals can be separated by multichannel system and array signal processing. However, multichannel system has the limitations of large volume and high cost, and cannot be used in some applications. For example, in satellite communication, due to the long transmission distance, the arrival direction difference of signals is small, so array signal processing cannot be used for separation, which requires single-channel system for separation. At present, digital mode is the main information unit in the network, and analog-to-digital conversion is the link that all the source information faces. After the system collects the information, it will encode or decode it according to the requirements of different network formats. Therefore, it is necessary to set up an audio and video compression encoder. In the secure data fusion method of industrial IoT, the fusion node refers to the node that fuses the information of nodes in the cluster [21]. Monitoring node refers to the common node established by the base station in the cluster or selected in four seasons, and its function is to ensure its reliability by monitoring the fusion information. In order to save the energy of sensor nodes, the nodes can be dormant when there is no need to collect data. The mobile collector can move randomly within and between subnets, and a fog server is installed on the mobile collector, thus forming a mobile fog node.

The article "Industrial Internet of Things Model Driven by Particle Filter and Network Communication Technology" was retracted in 2023. Reasons: signs of a paper mill; suspected computer-generated content; unreliable results or conclusions; concerns about the data.

### 3.2. Model Construction and Analysis

Filtering is to restore the real signal from the observed signal polluted by noise and try to eliminate or reduce the influence of noise on the original signal. The essence of filtering is actually statistical estimation. By combining the state prediction of the system with the observation, they can get the accurate estimation of the system state by iterative method. The main disadvantages of particle filter are weight degradation and sample exhaustion. Weight degradation means that the weights of most sampled particles tend to zero after repeated iterations, and only a few particles have larger weights, which will cause most of our computing resources to be wasted on most particles that have little effect on state estimation, with only a few particles that are valuable for state estimation. Although the introduction of resampling idea can effectively alleviate the degradation of particle weights, it also brings some problems such as sample exhaustion and increased calculation. In this paper, an improved particle filter algorithm is proposed to solve the problems of weight degradation and sample exhaustion of traditional particle filter. The network is based on the industrial sensor network. According to the actual needs, the sensor nodes will be deployed in different areas of the industrial site, and each area will form an interconnected subnet. However, there is a link reliability problem in the links between nodes, and the link reliability reflects the reliability of the links between nodes. It is related to the link quality between nodes, the sleeping mechanism of nodes, the remaining energy of nodes, and other factors. In signal processing problems such as communication, radar, biomedicine, etc., it is usually necessary to estimate the internal state of the system, but these states cannot be directly observed. Therefore, it is necessary to indirectly obtain the internal state information of the system by analyzing the external observations of the system. Such problems can be described by the following state space model:

(1) $$\begin{array}{c} \theta_{k}=f\left(\theta_{k-1},v_{k}\right), \end{array}$$

(2) $$\begin{array}{c} y_{k}=h\left(\theta_{k},n_{k}\right). \end{array}$$

Among them, *θ*_*k*_ is the *N*_*θ*_-dimensional state vector at the *t*_*k*_ moment; *y*_*k*_ is the *N*_*y*_-dimensional observation vector at the *t*_*k*_ moment; *v*_*k*_ and *n*_*k*_ represent the state transition noise vector and the observation noise vector, respectively. All sensor nodes use a simplified energy consumption model. According to this model, in the process of data forwarding, energy consumption consists of transmission energy consumption and reception energy consumption. The transmission energy consumption of *S*_*i*_ transmitting *B* bit data to *S*_*j*_ can be expressed as

(3) $$\begin{array}{c} E_{T}\left(i,j\right)=\left(E_{elec}+\varepsilon_{amp}d_{\left(i,j\right)}^{2}\right)B. \end{array}$$

The receiving energy consumption of *S*_*j*_ receiving *B* bit data can be expressed as

(4) $$\begin{array}{c} E_{R}\left(j\right)=E_{elec}+B, \end{array}$$

where *E*_*elec*_ represents the basic energy consumption per bit of data transmitted or received; *ε*_*amp*_ represents the energy consumption of the transmission amplifier; *d*_(*i*, *j*)_ represents the distance between *S*_*i*_ and *S*_*j*_. Therefore, the total energy consumption in the process of *S*_*i*_ transmitting *B* bit data to *S*_*j*_ can be expressed as

(5) $$\begin{array}{c} E_{R}\left(j\right)=E_{elec}+B. \end{array}$$

A special algorithm converts the actual information that was gathered into a code with no physical meaning, and this is referred to as a pattern in coding. In data fusion, the base station is in charge of the computation and generation of pattern codes; the fusion node only needs to map the pertinent data into the pattern codes. The data's confidentiality is somewhat ensured by mapping the gathered information into pattern code before transmission. At the same time, the fusion process is more effective and the computational overhead is lower due to the coding characteristics of the pattern code itself. The precision of the proposed distribution function will have a direct impact on the estimation of state. The following requirements should be met by a good importance density function: the support set range of the importance density function should include all positions in the posterior probability distribution; long tail should be present; it is essential to take into account the posterior distribution's effects from the transfer prior, likelihood probability distribution, and most recent observational data. The communication mechanism and server program flow of industrial IoT are shown in Figure 2.

The article "Industrial Internet of Things Model Driven by Particle Filter and Network Communication Technology" was retracted in 2023. Reasons: signs of a paper mill; suspected computer-generated content; unreliable results or conclusions; concerns about the data.

In this mechanism, the target monitoring probability is calculated first, and the communication radius of the target is obtained according to the distance information between the target and the node. On this basis, the next position of the target is calculated, the task allocation function is obtained, the constraint condition that a node can only join one cluster is given, and the balanced scheduling objective function of minimising the communication energy consumption between the target and the nodes in the cluster is calculated, so as to complete the balanced scheduling of the target tracking nodes in the IoT communication. If there is information missing at the node, first, intelligent scanning should be conducted to find out whether the surrounding environment has a coordinator. Then, the beacon is monitored within the scanning limit, so as to obtain the relevant information of the coordinator and send a connection request. Finally, the coordinator node is assigned a short URL, which contains the new address and the instruction of the connection success status, so that information communication can be carried out. The expected transmission energy consumption of each of the fog node's neighbours is determined, and the fog node with the lowest expected transmission energy consumption is chosen as the repeater when a node needs to choose a repeater to send data to a mobile fog node. The dual key of the base station is used to encrypt the data collected by the node before it is sent to the base station during the fusion stage. The base station then converts it into a pattern code and issues a signal indicating the correspondence between the data and the pattern code. The best method for balancing the scheduling of target tracking nodes in the Internet of Things chooses the initial optimal subset from among all nodes that are capable of perceiving target tracking and provides the balanced scheduling of target tracking nodes' objective function. The balanced scheduling of target tracking nodes for IoT communication is finished on this basis. Based on this, scheduling target tracking nodes in an optimal and balanced manner is an efficient way to address the aforementioned issues. The fog node will locally store the expected minimum energy consumption of the node and use it to determine which transponder to use for data transmission, thereby lowering the overall energy consumption of the data transmission.

For different particles of various discrete parts at *t* time, the approximate value of the posterior probability density can be calculated by the following formula:

(6) $$\begin{array}{c} f\left(\pi \left(X_{t}\right)=\rho |y_{1:t}\right)\approx \omega_{t}^{\left(i\right)}m_{\pi {\left(X_{t}\right)}^{\left(i\right)}}\left(\rho \right), \end{array}$$

where the attribution function is defined as

(7) $$\begin{array}{c} \int_{\partial }m_{\eta }\left(\ell \right)\delta \ell =\left\{\begin{array}{c} 1,\eta \in \partial ,\\ 0,\text{other}. \end{array}\right.. \end{array}$$

Classify all *π*(*X*_*t*_)^(*i*)^=*ρ* particles and calculate the probability, and then obtain the best estimate $\pi \left({\overset{\wedge }{X}}_{t}\right)$ of the discrete part *π*(*X*_*t*_) at the *t* moment according to the following formula:

(8) $$\begin{array}{c} \pi \left({\overset{\wedge }{X}}_{t}\right)=\arg\underset{\rho }{\max}f\left(\pi \left(X_{t}\right)=\rho |y_{1:t}\right). \end{array}$$

When an estimate of the discrete part is obtained, an estimate of the magnitude can be obtained by Kalman filtering. For any node *S*_*i*_ within the data collection range, the expected minimum energy consumption is

(9) $$\begin{array}{c} EMC\left(i\right)=\left\{\begin{array}{c} \left(2\left\lfloor h_{0}\right\rfloor \right)E_{elec}B+\frac{\varepsilon_{amp}d_{\left(i,i+h\right)}^{2}B}{\left\lfloor h_{0}\right\rfloor },\\ \left(2\left\lceil h_{0}\right\rceil \right)E_{elec}B+\frac{\varepsilon_{amp}d_{\left(i,i+h\right)}^{2}B}{\left\lfloor h_{0}\right\rfloor }. \end{array}\right.. \end{array}$$

Among them,

(10) $$\begin{array}{c} h_{0}=\sqrt{\frac{\varepsilon_{amp}}{2E_{elec}}}d_{\left(i,i+h\right)}. \end{array}$$

In order to obtain the minimum energy consumption of *S*_*i*_ to forward the *B* bit data to the mobile node, it is assumed that *S*_*i*_ can forward the *B* bit data to the mobile node along a path of *h* hops.

The article "Industrial Internet of Things Model Driven by Particle Filter and Network Communication Technology" was retracted in 2023. Reasons: signs of a paper mill; suspected computer-generated content; unreliable results or conclusions; concerns about the data.

Not only should a good resampling algorithm minimise the degradation of particle weights, but also it should maximize the diversity of the particles and minimise the algorithm's execution time. This paper considers that the process of data forwarding to a mobile node can be divided into two processes for any node that is not within the one-hop range of the mobile node in order to make the measurement of expected transmission energy consumption more thorough for the measurement of a node's data forwarding capability. Specifically, it does this by sending data to its neighbours, who then sends it to the mobile fog node. Other servers in the server group should be chosen to send the cached data if more replies are sent than the allowed limit. The transmission of wireless signals should be carefully considered due to the large number of nodes in various information transceivers, and the reliability of information transmission can be ensured by using the network topology of ZigBee wireless sensor devices to forward information to nodes. The fusion node and the monitoring node are chosen simultaneously based on the clustering algorithm to take advantage of the robustness and adaptability of the monitoring mechanism, reduce unnecessary communication overhead, and enhance the network's robustness and the data's freshness.

## 4. Result Analysis and Discussion

In order to verify the rationality of the communication mechanism design of industrial IoT based on particle filter and the performance of the algorithm, experiments are carried out in this chapter. The monitoring standards are systematically constructed, the hardware and software functions are tested, and the results are properly analyzed. In order to prove that the improved particle filter algorithm can better estimate the channel, the sum-sum least mean square estimation and least square estimation methods are introduced in the experiment. Energy consumption is defined as the energy consumed by the source node in the process of forwarding data to the fog node. To evaluate the energy consumption performance of the proposed algorithm, a 400 m × 400 m subnet is selected. The long communication radius of the mobile fog node is 120 m. The energy threshold of a node is 25%. Firstly, the circuit of information intelligence running state is detected, and each wireless communication technology module is connected with information intelligence. The breakdown state of the monitor needs to be adjusted according to different information; otherwise the system monitoring effect will be inaccurate. The sample of channel estimation is shown in Figure 3.

The results show that the improved algorithm has better estimation quality than the original algorithm. In the IoT environment, the data of real-time wavelengths of different information quantities and one information wavelength are shown in Table 1.

This mechanism can effectively collect the sensor data of industrial field and analyze and process the sensor data by using the architecture, which will finally help improve the industrial field application. In addition, the method does not need a large number of operators to participate, thus reducing the labor cost and further reducing the production cost of enterprises.  Figure 4 shows the MSE (mean square error) curve of the residual noise in the estimated value of the source signal.

The experimental results further confirm the effectiveness and practicability of applying the particle filter algorithm in industrial IoT communication. The calibration accuracy of the wavelength coefficient of information transmission in the intelligent information monitoring system of IoT communication terminal largely determines the monitoring accuracy of the monitoring system. Therefore, this paper synthesizes the wavelength coefficient of the whole information to minimise the system error, so as to quickly improve that accuracy of intelligent information monitor by the monitoring system, ensure the monitor accuracy, and promote the monitoring effect to be higher and the system to be stable. The signal detection performance of different algorithms is shown in Figure 5.

The article "Industrial Internet of Things Model Driven by Particle Filter and Network Communication Technology" was retracted in 2023. Reasons: signs of a paper mill; suspected computer-generated content; unreliable results or conclusions; concerns about the data.

Although 180-degree phase ambiguity sometimes appears in channel estimation, due to the introduction of differential encoding/decoding operation, the phase ambiguity will not affect the signal detection performance, which is proved by the low bit error rate characteristic shown in Figure 5.  Table 2 shows the energy consumption of different algorithms.

It can be seen that the energy consumption increases with the increase of node density. This is mainly because the expansion of network density not only improves network connectivity, but also increases the number of neighbours of nodes, which makes nodes have more choices when looking for repeaters, which increases the number of hops of data forwarding paths from source nodes to fog nodes, thus increasing energy consumption.  Figure 6 shows the comparison of simulation running time of different algorithms.

Aiming at the shortcomings of traditional particle filter algorithm, this paper proposes an improved algorithm to better solve this problem. The results show that the running time of this algorithm is short, and the results also prove the efficiency of this improved algorithm.  Figure 7 shows the accuracy comparison of the algorithm.

It can be seen that, with the increase of the number of experiments, the accuracy of the algorithm is stable at about 95%, and the real-time wavelength tends to be stable. Comparing the accuracy of the improved algorithm with that of the traditional algorithm, the accuracy of the improved algorithm is much higher than that of the traditional algorithm.

In this chapter, many experiments are carried out to verify the performance of the improved algorithm. The results show that the accuracy rate of the proposed algorithm is 95.54%, which is higher than that of the comparison algorithm. At the same time, the improved algorithm proposed in this paper can obtain better parameter estimation performance and realise signal separation with low bit error rate. This shows that the algorithm proposed in this paper has superior performance. The experimental results further confirm the effectiveness and practicability of applying the particle filter algorithm in the communication mechanism of industrial IoT.

The article "Industrial Internet of Things Model Driven by Particle Filter and Network Communication Technology" was retracted in 2023. Reasons: signs of a paper mill; suspected computer-generated content; unreliable results or conclusions; concerns about the data.

## 5. Conclusions

Particle filtering converts the high-dimensional integral in Bayesian estimation into a multiplication and accumulation operation in order to approximate the real posterior distribution of the state using the weighted sum of a collection of random samples from the posterior distribution of the state to be estimated. This processing technique is applicable to any nonlinear, non-Gaussian model and is not constrained by the system model. However, the conventional particle filter has some drawbacks, including sample exhaustion and weight deterioration. The traditional multiuser detection method has some limitations in terms of practical application because it typically assumes that the number of active users is constant during the communication process. In this paper, a particle filter-based industrial IoT communication mechanism and algorithm are presented. A mobile collector with a server is used as a mobile node in this mechanism to collect data. The node uses the suggested routing mechanism based on anticipated transmission energy consumption to forward the perceived data to the node during data collection. The system is advanced and useful because it uses the network server to connect the client and database at the same time. After the data has been collected, the nodes categorise it. Some of the data is then processed locally, while the remainder is uploaded to the cloud, enabling reasonable use of the cloud architecture to realise the efficient analysis and processing of the data. Several experiments were conducted to confirm the effectiveness of the improved algorithm in this paper. The outcomes demonstrate that the algorithm suggested in this paper performs better. The proposed algorithm's accuracy rate is 95.54 percent, higher than the comparison algorithm's. Additionally, the enhanced algorithm suggested in this paper can achieve signal separation with a low bit error rate and improve parameter estimation performance. The experimental findings support the usefulness and viability of using the particle filter algorithm in the industrial IoT's communication system. The approach outlined in this paper is workable. However, there are still a lot of issues that need to be studied in this paper due to the limited level of personal knowledge and the lack of writing time. The universally applicable particle filter dimension reduction technology will be looked at in more detail in the following step.

## Figures and Tables

**Figure 1:** Layering and application model of IoT.

**Figure 2:** Communication mechanism and server program flow of industrial IoT.

The article "Industrial Internet of Things Model Driven by Particle Filter and Network Communication Technology" was retracted in 2023. Reasons: signs of a paper mill; suspected computer-generated content; unreliable results or conclusions; concerns about the data.

**Figure 3:** Sample of channel estimation.

**Figure 4:** MSE curve of residual noise in the estimated value of source signal.

**Figure 5:** Signal detection performance of different algorithms.

**Figure 6:** Comparison of simulation running time of different algorithms.

**Figure 7:** Accuracy comparison of algorithms.

**Table 1:** Information wavelength data of communication terminal information intelligent monitoring system.

Information quantity	Real-time wavelength/nm	Single information wavelength/nm	Information wavelength coefficient/nm
1	1456.131	1456.132	92.984
5	1456.179	1456.132	93.014
10	1456.254	1456.132	93.187
20	1456.978	1456.132	94.752
40	1457.342	1456.132	95.468
60	1458.287	1456.132	96.017
100	1460.241	1456.132	97.354

**Table 2:** Energy consumption of different algorithms.

Number of nodes	POFA algorithm	ExOR algorithm	Improved algorithm in this paper
800	0.351	0.236	0.197
900	0.356	0.243	0.199
1000	0.462	0.248	0.204
1100	0.517	0.251	0.209
1200	0.628	0.257	0.213

## Data Availability

The data used to support the findings of this study are available from the corresponding author upon request.
